# Strategies to Improvise Organ Donor Pool: A Study on the Knowledge, Attitudes, and Performance of Higher Secondary School Teachers Towards the Organ Donation

**DOI:** 10.1155/2022/5438492

**Published:** 2022-06-28

**Authors:** Krishnaraju Venkatesan, Durgaramani Sivadasan, Neelaveni Thangavel, Shadia Hamoud Alshahrani, Premalatha Paulsamy, Kandasamy Muthugounder, Kousalya Prabahar, Gamal Osman Elhassan, Kalpana Krishnaraju, Sirajudeen SheikhAlavudeen, Kumar Venkatesan, Kenenisa Dekeba

**Affiliations:** ^1^Department of Pharmacology, College of Pharmacy, King Khalid University, Abha, Asir, Saudi Arabia; ^2^Department of Pharmaceutics, College of Pharmacy, Jazan University, Jizan, Saudi Arabia; ^3^Department of Pharmaceutical Chemistry, College of Pharmacy, Jazan University, Jizan, Saudi Arabia; ^4^College of Nursing, Mahalah Branch for Girls King Khalid University, Asir, Saudi Arabia; ^5^Dharan Nursing College, Salem, Tamilnadu, India; ^6^Department of Pharmacy Practice, Faculty of Pharmacy, University of Tabuk, Tabuk-71491, P .O. Box-741, Saudi Arabia; ^7^Department of Pharmaceutics, Unaizah College of Pharmacy, Qassim University, Alqassim, KSA, Saudi Arabia; ^8^Department of Pharmaceutical Chemistry &Analysis, School of Pharmaceutical Sciences, Vels Institute of Science, Technology and Advanced Studies (VISTAS), Chennai, India; ^9^Department of Pharmaceutics, Faculty of Pharmacy, Omdruman Islamic University, Omdurman, Khartoum, Sudan; ^10^Department of Clinical Pharmacy, College of Pharmacy, King Khalid University, Abha, Saudi Arabia; ^11^Department of Pharmaceutical Chemistry, College of Pharmacy, King Khalid University, Asir-Abha, Saudi Arabia 61421; ^12^Department of Food Process Engineering, College of Engineering and Technology, Wolkite University, Wolkite, Ethiopia

## Abstract

**Introduction:**

This study aimed to assess higher secondary school teachers' knowledge, attitude, and performance levels towards organ transplantation and donation (OTD). Teachers have an essential role in giving knowledge to children and teenagers, and they can influence their views. Organ transplantation offers re-life to many patients, yet organ shortages are a global issue. Teachers who influence students' future attitudes regarding organ donation must have a favorable attitude and genuine knowledge.

**Materials and Methods:**

The research method was descriptive and cross-sectional. The sample size was 372 school teachers in Villupuram district of Tamilnadu, India, selected using a convenient sampling method. A survey questionnaire was used to assess the knowledge and attitude about OTD, the reason for donating/not donating organs. Multivariate analysis was performed to identify critical variables affecting intent to practice.

**Results:**

The teachers' mean scores with SD on knowledge, attitude, and performance were 7.61 ± 2.74, 8.81 ± 2.08, and 0.38 ± 0.11, respectively. The linear regression analysis showed that the knowledge (*p* < 0.001) and attitude (*p* < 0.05) of the participants were positively associated with organ donation performance. A significant relationship was also observed between gender (*p* < 0.036), age (*p* < 0.01), and education status (*p* < 0.001) with the performance of the teachers. Lack of family support was the most spelt reason for unwillingness for organ donation.

**Conclusion:**

The positive linear correlations underline that having more information may lead to a more optimistic mindset and, as a result, to better practices. Teachers should be provided with overall health teaching campaigns to increase the number of possible organ donors. Teachers serve as role models for students, families, and society by changing their attitudes.

## 1. Introduction

Organ transplantation can save the lives of people suffering from end-stage organ disease. Organ transplants have been performed on men, women, and children of different ages, nationalities, and walks of life [1]. Every year, almost 500,000 people die in India due to a lack of organs, partly due to the country's small number of organ donors [2]. According to 2016 figures, India has a 0.34 per million population rate of dead donor transplantation [3].

Organ transplantation provides a life-saving opportunity for those patients with the end-stage organ-specific disease. Men, women, and children of all ages, ethnicities, and walks of life have had organ transplantations [1]. In India, nearly 500,000 people die every year because of the non-availability of organs [4], primarily attributed to a limited number of organ donors [3]. According to 2016 statistics, India showed a deceased donor transplantation rate of 0.34 per million population [4]. Compared to Europe's 21.53 deceased organ donors per million population, this figure is relatively low [5]. This may be due to a lack of education and awareness regarding organ donation, religious attitudes, and superstitious beliefs, which have caused dread and mistrust among the general public [6, 7].

Despite a rise in living donor transplant activity over the previous two decades, with 6772 kidneys and 1313 livers transplanted in India in 2018, the real demand is predicted to be 12,578 kidneys and 4173 livers yearly (as reported to National Organ and Tissue Transplant Organization, 2018) [8]. In this context, the Tamil Nadu state in India has a good record of organ donation, with 1.3 donor pmp (per million population) [9]. According to an educational program launched by an organ procurement group, a multipronged strategy is needed to enhance organ donation. According to the findings of research done by Sadic et al., there is a need for more coordination between religious authorities, healthcare professionals, and school instructors to lessen the enormous gap between the supply and demand of organs for transplantation [10].

According to the findings of a research conducted by Febrero et al. in Spain, 75% of teachers support organ donation, and psychological variables impact their attitudes [11]. Furthermore, the findings of Roeyzet al. revealed that teachers' awareness of brain death has a favorable impact on their views regarding organ donation, and given that teachers are community educators, training is required to improve their knowledge level in this area [12]. It should be mentioned that the majority of instructors and students support the school's organ donation curriculum and that kids' education at school has an impact on families' attitudes toward organ donation [13]. Furthermore, Khaddami et al. found that the primary reasons for instructors not participating in the organ donation procedure were lack of awareness about chronic illness patients and a lack of faith in the organ transplant system. As a result, instructors must develop confidence in brain death diagnosis tools and suitable teaching activities [14].

After the Sydney Declaration in 1968 [15], the idea and knowledge of brain death became widely recognized. Many nations began their programs in the early 1970s by establishing the legal framework required to verify brain death, followed by donating organs. The Transplantation of Human Organs Act (THOA) of 1994, as amended in 2011 and rules issued in 2014, establishes the legal framework for brain death and organ donation in India [16]. This act developed a clear and reliable framework to assist India's urgent demand for organ transplantation. While several non-governmental organizations, such as the MOHAN foundation, and individuals worked hard to raise awareness, the much-needed boost came in the form of concrete steps taken by state governments of India, such as Tamil Nadu [17, 18], which were later followed by Karnataka, Maharashtra, Kerala, and others. The National Organ and Tissue Transplant Organization were founded to oversee the whole program under the direction of India's Ministry of Health. The much-needed drive for any program's success comes only when top management advocates for it. In just a few years, India's organ donation rates jumped from a pitiful 0.05 pmp to a whopping 0.8 pmp [19].

Teachers' information and knowledge build the foundation for students' future attitudes on this subject. As a result, it is critical to know what instructors know about brain death and organ donation. A few studies on patients, their families, and healthcare personnel have also been conducted [20, 21]. However, studies on populations with a better chance of addressing the present organ donor shortage have yet to be conducted. The current research examines higher secondary school teachers' knowledge, attitudes, and beliefs about organ donation, as well as the factors that influence their desire to give organs in South India. The findings imply that an environment conducive to organ donation might be established by raising understanding and removing some unfavorable attitudes among instructors. This might increase the number of people who register as organ donors and donate organs each year. This needs more interventional investigations to validate the findings.

## 2. Methods

### 2.1. Design

The current study is a descriptive cross-sectional survey on teachers working in male and female elementary and secondary schools in the Villupuram district, Tamilnadu, India.

### 2.2. Population and Setting

Teachers working in male and female secondary schools in the Villupuram district were the study's target population. The Villupuram educational district had 2897 functioning schools, among which 289 schools were offering higher secondary education. These schools were distributed in 5 blocks, and 372 school teachers were selected randomly out of 961 from the 289 higher secondary schools (Figure 1).

### 2.3. Sample Size and Sampling Process

According to Raosoft's online sample size calculator, the minimum recommended sample size was 277, with a 95% confidence level, 50% response rate, and a 5% margin of error. In this study, 372 teachers (192 female, 180 male) were selected to improve the generalization of the results.

### 2.4. Data Collection Tools/Instruments

This study used a prestructured, pretested questionnaire on various aspects of organ donation. The individual questionnaire consists of 36 questions pertaining to demographics (3 questions), knowledge (12), attitude (7), the reasons for not donating organs (7) and reasons for donating organs (5), and performance (3). The knowledge section questions had three answers, yes (1 point), no (0), and not sure (0), and the total score for this section was 12. Scores less than ≤4 were considered the poor level of knowledge, scores between 5 were regarded as moderate level of knowledge, and scores greater than eight were considered a good level of knowledge. The attitude questionnaire was graded on a Likert scale from agree (3 points), do not know (2 points), and disagree (1 point) with a total score of 21. Scores ≤7 were considered poor, scores between 8 and 14 to have a moderate attitude, and scores >15 to have a good attitude. The attitude was further assessed by asking why not donating organs (7) and the reason for donating organs (5). In this section, if ‘yes”3', ‘no' ‘1' and for ‘not sure' ‘2' grades were given for reason for donation and reverse score was given for not donating organ section. The higher score indicated a good attitude. The performance criteria included having a history of receiving or donating an organ, having a donation card or processing for a donation card, encouraging others to donate, or being willing to donate an organ in the event of need. Positive responses received one point, while negative reactions received zero, for a total score of three. One was rated as poor, two as moderate, and three as excellent. The questionnaire's content validity was obtained by a review of 8 corresponding experts in medicine and healthcare. The Cronbach's alpha coefficient was 0.83 for the entire questionnaire.

### 2.5. Ethical Consideration

Official permission to conduct the study was obtained from the Director, Directorate of Education, Villupuram district, and Head of the Institution of all the schools selected for the study. Additionally, written consent from the participants was collected before starting the study after explaining the aim of the study, their role, the confidentiality of the information, and their right to depart from the study at any point of data collection. Ethical approval was obtained from the Institutional Ethical Committee with ICE/LCN/2021-11 dated 20.10.2021.

### 2.6. Statistical Analyses

The data was processed and analyzed by SPSS software using descriptive and inferential statistics. Descriptive statistics, Student *t-*test, *χ*^2^ tests (for categorical variables), and regression analysis were used. Regression analysis is used to estimate the relationships between performance, knowledge, attitude, and demographics of the participants.

## 3. Results

Among the overall respondents, 365 (*n*), 188 (51.5%) were male, and 177 (48.5%) were female. The majority of the participants were above the age of 35 years. The respondents predominantly held a postgraduate qualification (95.6%) (Table 1).

After completing the questionnaire, it was discovered that 100% claimed that they were aware that organs could be given to save another person's life. Only 3.3% (*n* = 12) had completed an organ donation card. Nearly 41% (*n* = 150) of the instructors believe that giving organ donation poses a danger to the donor's health. According to the majority of instructors, we should not sell the organs (*n* = 222, or 61%). Many of the instructors (65.8%) were aware that there is a legislative statute considers brain death as a kind of death in India, allowing organs such as kidneys, hearts, livers, and lungs to be given to patients in need.

Nearly 47% (*n* = 170) were aware, and the remaining participants were not aware or not sure that it is illegal for donors or their families to accept monetary or other benefits from the recipient for organ donation in India. Most favorably, all participants agreed that they heard of brain death. But, many participants were not familiar with organ donor cards as 71.2% (260) and only 3.3% (12) owned the card. A more significant number of participants, 245 (67.1%), know that one can donate their organs while living and even after death.

Regarding the organs that can be donated while living, many participants showed positive knowledge for kidney (57.5%), liver (48.7%), and skin (70.7%) while reduced response for lung (29%), intestines (28.2%), and pancreas (7.7%). All participants expressed a clear idea about the donation of heart and cornea. Major participants (68.2%) were not clear about the state-run organization that coordinates and supervises deceased donor and living donor transplant activities, including transparently distributing organs by maintaining an online waitlist registry (Table 2).

### 3.1. Attitude

Of all the respondents who took the survey, 51% said that for the next of kin, they were not willing to consider organ donation of a relative in the event of brain death compared to 32% of the respondents who were willing to do so. Around 79.2% (*n* = 289) of participants do not have any experience donating their relative's organs. Half of the participants (51.7%) (*n* = 189) showed interest to donate their organs, and nearly similar proportions (49.9%) (*n* = 182) were interested in donating their organs to an unknown person. Seventy-four percent of participants (*n* = 270) think that educational program related to organ donation and transplantation is required for higher secondary school students. Nearly equal proportions of participants (41.6 vs 45.8%) liked and disliked applying for donor cards. But, 85.5% (*n* = 312) of participants responded positively to own a donor card if they receive more information on organ donation (Table 3).

### 3.2. Reasons for Refusal of Organ donation

The majority of participants (27.5%; *n* = 46) who refused organ donation felt that their family might not support their decision to donate organs (Table 4). Others (11.5%; *n* = 42) expressed concerns that their organs will not go to those patients who need them most.

### 3.3. Reasons for Willingness to Donate Organs

The reasons for consent to organ donation are shown in Table 5. More than half of the participants (*n* = 106, 63.5%) expressed their sense of organ donation as the desire to help others. A part of the participants (*n* = 42, 11.5%) was willing to donate organs, as the organs would have no use to the donor once dead. A few (*n* = 31, 8.5%) was moved by the importance of transplantation in saving lives.

### 3.4. Performance

A checklist assessed the performance of the teachers with three questions such as (1) having a history of receiving or donating an organ, (2) having a donation card or processing for donation card, and (3) encouraging friends, family and others to donate an organ in the event of need. The teachers' mean scores on knowledge, attitude, and performance with SD are 7.61 ± 2.74, 8.81 ± 2.08, and 0.38 ± 0.11, respectively. Among the three variables studied, though the level of performance was inferior, the positive linear correlations (Table 6) reaffirm that more knowledge can lead to a more positive attitude and, as a result, to better practices.

### 3.5. Multivariate Analysis

According to Table 7, the knowledge level (*p* = 0.001) and attitude (*p* = 0.05) of the participants were positively associated with the participants' performance on organ donation. A significant relationship was also observed between gender (*p* = 0.036), age (*p* = 0.01), and education status (*p* = 0.001) with the performance of the participants.

## 4. Discussion

The present study shows that a maximum number of teachers (65.8%) were aware that organ donation is regulated by law in India, and there is a need to make these laws more effective. Similar findings were found in many studies [22–24] and to mention one, a study conducted by Bharambe et al., in the Konkan region of Maharashtra, among the rural community, which showed that 67.2% of respondents were aware that there is legislation related to organ donation [25]. Most of the participants were aware that it is illegal for donors or their families to accept monetary or other benefits from the recipient for organ donation in India. In a study conducted by Vijayalakshmi et al., in Karnataka, among the general population, it was observed 87% of subjects were aware that selling organs is illegal in India [26]. This increased knowledge among people may be due to recent efforts by the regulatory authorities to understand organ donation.

In contrast to the knowledge level, only 51.7% of the participants were interested in donating their organs. The knowledge level does not go with attitude hand in hand. Based on these study results, to see a change in society, the government and other aided organizations working on this organ donation segment should focus on people's attitudes more than enhancing knowledge. Surprisingly, when a question was asked to teachers, whether they would be interested in registering for a donor card if they were given more factful information about the importance of organ donation, 85.5% showed a positive response. This implies positive psychology of the participants that they might agree for a positive change if they were convinced. Another hindrance in organ donation, while a person is on brain death, is, next to kin has to sign the acceptance for organ donation. In this study, only 32% were willing to sign for their relative. This highlights the importance of registering for a donor card and the knowledge for avoiding emotional hindrance. Significantly, teachers should be appraised for taking self-initiative to counsel their relatives or unknown person about the importance of organ donation.

According to the present study, most of the study participants, that is, 74% of teachers, believe that organ donation should be made a part of the curriculum. Such a large number indicates that they understand the importance of organ donation and realize that educational intervention is necessary to increase their knowledge about donating organs.

The current survey intended to understand the hindrance among the teachers for refusing organ donation. Despite the highly educated community, most participants (27.5%) refused because their family may not support their decision to donate organs. Again, this emphasizes the social and emotional hindrance even among the educated peoples and the need to focus on this public behavior to bring about the required positive knowledge. Few participants (11.5%) were hesitant because their organs would not go to those patients who need them most, and some worried that donating organs would disfigure their bodies. This again attracts the level of transparency required in the entire process, and the need for an educational program to address this aspect more clearly to the participants and the general public. Devi et al. observed that 26% of people were afraid of mutilation, which supports the findings of this study [27]. According to research by Srinivasula et al., nearly two-thirds of pupils in Hyderabad were afraid of being disfigured [28]. It was also one of the critical reasons for organ donation not being popular in India, according to a study done by Sugumar et al. [29]. The fear of physical deformity following organ retrieval is a significant barrier that prevents individuals from giving organs.

More interestingly, the majority of the participants (63.5%) agreed to donate organs with the desire to help others. Humanity is still alive. Coinciding with this intention, 11.5% of participants agreed to contribute, as they considered that the organs have no use to the donor after death. Similar to the above attitude, 8.5%was moved by the importance of transplantation in saving lives.

Unfortunately, compared to the general population's perceptions of organ donation toward improving the supply of organs, very little has been published about teachers' attitudes towards organ donation. We recommend further widespread educational and motivational programs regarding deceased organ donation in educational institutions as the positive attitude of faculty is vital for students as they spend maximum time in schools and colleges. Further studies should be conducted to evaluate the effectiveness of this type of educational program on other larger populations.

### 4.1. Clinical Significance

School teachers should have a thorough knowledge and favorable attitude towards organ donation and be the role models to future generations. They can be the “change agents or catalysts” among the students and society to inculcate appropriate knowledge and a positive attitude to them from an early stage. “Catch them Young” is the saying that will be the best-suited phrase for the school children, and for this, the teachers will be the best choice.

## 5. Conclusion

According to the findings of this study, teachers' awareness, attitude, and performance concerning organ donation are interrelated with each other and to their demographic characteristics like gender, age, and qualification. The positive linear correlations reaffirm that more knowledge can lead to a more positive attitude and, as a result, to better practices. Hence, educational interventions should be targeted to the teachers to educate and motivate the students and community to provide full support to those who wish to donate organs.

## Figures and Tables

**Figure 1:** Flow chart.

**Table 1:** Gender, age, and education distribution of the respondents (*n* = 365).

Demographic variables	n	%
Male	188	51.5
Female	177	48.5
Age (years)		0
<35	121	33.2
35-50	144	39.5
>51	100	27.4
Educational qualifications		
Post graduation	349	95.6
PhD	16	4.4

**Table 2:** Knowledge about organ donation and brain death.

S.no	Questions	Response					
		Yes		No		Not sure	
		*n*	%	*n*	%	*n*	%
1	Are you aware that organs can be donated to save another person's life?	365∗	100	0	0	0	0
2	Do you think living organ donations involve any health risks for the donor?	150	41.1	125	34.2	90	24.7
3	Can we sell our organs (like kidneys)?	45	12.3	222	60.8	98	26.8
4	Are you aware that a parliamentary law in India recognizes brain death as a form of death so that organs like kidneys, heart, liver, and lungs can be donated to needy patients?	240	65.8	54	14.8	81	240
5	Concerning organ donation in India, is it illegal for donors or their families to accept monetary or other benefits from the recipient?	170	46.6	61	16.7	134	36.7
6	Have you heard of brain death?	365	100	0	0	0	0
7	Do you know what an organ donor card is?	46	12.6	260	71.2	59	16.2
8	Do you own an organ donor card?	12	3.3	296	81.1	57	15.6
		Response					
9	When do you think one can donate their organs?	During life		After death		Both	
		52	14.2	34	9.3	245	67.1
		Response					
10	When do you think the following organs can be donated?	Living donation		Deceased donation		Not sure	
	Kidneys	210	57.5	133	36.4	22	6
	Liver	178	48.8	63	17.3	124	34
	Skin	258	70.7	98	26.8	9	2.5
	Lung	106	29	81	22.2	178	48.8
	Intestines	103	28.2	88	24.1	174	47.7
	Pancreas	28	7.7	149	40.8	188	51.5
	Heart		0	365	100		0
	Cornea		0	365	100		0
		Response					
		*n*	%				
11	Which state-run organization in Tamil Nadu coordinates and supervises deceased donor and living donor transplant activities, including distributing organs in a transparent manner by maintaining an online waitlist registry?		0				
	NOTTO	21	5.8				
	MOHAN foundation	86	23.6				
	ORGAN India	0	0				
	TRANSTAN	9	2.5				
	GIFT organ	0	0				
	Not clear	249	68.2				

**Table 3:** Attitude towards organ donation and donor card.

Questions	Response					
	Agree	%	Not agree	%	Do not know	%
1. Would you be willing to donate the organ(s) of a brain dead relative for the next of kin?	117	32	186	50.9	62	16.9
2. Do you have a relative whose organs have been donated?	58	15.8	289	79.2	18	4.9
3. Would you like to donate your organs?	189	51.7	112	30.7	64	17.5
4. Will you be interested in donating your organs to an unknown person?	182	49.9	114	31.2	69	18.9
5. Do you think an organ donation and transplantation educational program is required for higher secondary school students?	270	74	81	22.2	14	3.8
6. Do you like to apply for a donor card?	152	41.6	167	45.8	46	12.6
7. Do you think, if you receive more information on organ donation, it will support you for owning a donor card?	312	85.5	37	10.1	16	4.4

**Table 4:** Reasons for refusal of organ donation or applying for a donor card.

Statements	Response	
	n	%
1. I feel my family may not support my decision to donate my organs	46	27.5
2. I have concerns that my organs be used for medical research rather than for patients	21	5.8
3. I have concerns that my organs will not go to those patients who need them most	42	11.5
4.I feel like I am too old to donate my organs	7	1.9
5. I feel my medical comorbidities prevent me from donating my organs	12	3.3
6. I feel the surgery for donating organs will disfigure my body	18	4.9
7.Not sure	21	5.8

**Table 5:** Reasons for organ donation or applying for a donor card.

Statements	Response	
	*n*	%
1. Desire to help others	106	63.5
2. Personal experience with organ donors/recipients	4	1.1
3. Believing organs would have no use to the donor once dead	42	11.5
4. The importance of transplantation in saving lives	31	8.5
5. None of the above	6	1.6

**Table 6:** Correlation between knowledge, attitude, and performance of the teachers on organ donation.

Variable	Correlation coefficient	*p* Value∗
Knowledge-attitude	0.21	<0.05
Knowledge-practice	0.42	<0.05
Attitude-practice	0.33	<0.05

∗Correlation significant at 0.05 level (2-tailed).

**Table 7:** Regression analysis of performance with knowledge, attitude, and selected participant characteristics.

Variables	Beta coefficient	*t* Value	*p* Value	95% CI	
				Lower	Upper
Knowledge	0.19	4.7	0.001	0.23	0.6
Attitude	0.31	2.71	0.05	1.51	2.27
Gender	0.28	2.31	0.036	1.86	2.06
Age	0.71	3.9	0.01	0.09	0.32
Education	0.49	5.18	0.001	0.26	0.52

## Data Availability

The datasets used and/or analyzed during the current study are available from the corresponding author on reasonable request.

## Additional Points

*Institutional Review Board Statement.* Institution Ethical Committee gave an ethical clearance with ICE/LCN/2021-11 dated 20.10.2021.

## References

[1] Milaniak I., Wilczek-Rużyczka E., Wierzbicki K., Sadowski J., Kapelak B., Przybyłowski P. (2016). Evaluation of the motivation to consent to and to refuse organ donation among participants of educational meetings concerning organ transplantation. *Transplantation Proceedings*.

[2] Mithra P., Ravindra P., Unnikrishnan B. (2013). Perceptions and attitudes towards organ donation among people seeking healthcare in tertiary care centers of coastal South India. *Indian Journal of Palliative Care*.

[3] Abraham G., Vijayan M., Gopalakrishnan N. (2016). State of deceased donor transplantation in India: a model for developing countries around the world. *World Journal of Transplantation*.

[4] Ahuja A. (2017). Lack of organ donation in India: here is why half a million people die annually in India due to unavailability of organs. *NDTV*.

[5] The Council Of Europe European Committee (Partial Agreement) (2017). On Organ Transplantation. *NEWSLETTER TRANSPLANT International figures on donation and transplantation*.

[6] Spencer M. (2012). The barriers to organ and tissue donation in palliative care. *End of life journal*.

[7] Reddy A. V. R., Guleria S., Khazanchi R. K., Bhardwaj M., Aggarwal S., Mandal S. (2003). Attitude of patients, the public, doctors, and nurses toward organ donation. *Transplantation Proceedings*.

[8] Global Observatory on Donation and Transplantation (GODT) http://www.transplant-observatory.org/summary/.

[9] Abraham G., Reddy Y. N., Amalorpavanathan J. (2012). How deceased donor transplantation is impacting a decline in commercial transplantation: the Tamil Nadu experience. *Transplantation*.

[10] Sadic S., Sadic J., Krupic R., Fatahi N., Krupic F. (2016). The influence of information and religion on organ donation, as seen by school teachers in Bosnia and Herzegovina. *Materia socio-medica*.

[11] Febrero B., Ríos A., López Navas A. (2014). A multicenter study of the attitude of secondary school teachers toward solid organ donation and transplantation in the southeast of Spain. *Clinical Transplantation*.

[12] Ríos A., Febrero B., López-Navas A. (2012). Knowledge of the brain-death concept among secondary school teachers. *Transplantation Proceedings*.

[13] Siebelink M. J., Verhagen A. A. E., Roodbol P. F., Albers M. J. I. J., Van de Wiel H. B. M. (2017). Education on organ donation and transplantation in primary school; teachers' support and the first results of a teaching module. *PloS one*.

[14] Khoddami-Vishteh H. R., Ghorbani F., Ghasemi A. M., Shafaghi S., Najafizadeh K. (2011). Attitudes toward organ donation: a survey on Iranian teachers. *Transplantation proceedings*.

[15] Gilder S. S. (1968). Twenty-second world medical assembly. *British Medical Journal*.

[16] National Organ Transplant Program *Director General of Health Services India*.

[17] TRANSTAN-Transplant Authority of Tamil Nadu: Cadaver Transplant Programme Government of Tamil Nadu: Tamil Nadu Network of Organ Sharing. https://www.transtan.org.

[18] Shroff S. (2009). Legal and ethical aspects of organ donation and transplantation. *Indian journal of urology: IJU: journal of the Urological Society of India*.

[19] Pandit R. A. (2017). Brain death and organ donation in India. *Indian Journal of Anaesthesia*.

[20] Mohammadpour M., Mohammadpour A., Ajam-Zibad H., Najafi S. (2018). A study on the awareness, attitudes and performance of teachers towards the organ donation during 2016-2017. *Nursing Practice Today*.

[21] Alex A., Shroff S., Paul V. B. (2019). Did an increase in knowledge and awareness about organ donation improve organ donation rate in India over the past two decades?. *Indian Journal of Transplantation*.

[22] Nallusamy S., Shyamalapriya B., Ranjan Y. (2018). Organ donation – Current Indian scenario. *Journal of the Practice of Cardiovascular Sciences*.

[23] ROAD ACCIDENTS IN INDIA (2017). Road Accidents in India. *Transport research wing*.

[24] Srivastava A., Mani A. (2018). Deceased organ donation and transplantation in India: promises and challenges. *Neurology India.*.

[25] Bharambe V. K., Arole V. U., Puranam V., Kulkarni P. P., Kulkarni P. S. (2018). Knowledge and attitude toward organ donation among health-care professionals in a rural town in India. *Saudi Journal of Kidney Diseases and Transplantation*.

[26] Vijayalakshmi P., Sunitha T. S., Gandhi S., Thimmaiah R., Math S. B. (2016). Knowledge, attitude and behaviour of the general population towards organ donation: an Indian perspective. *National Medical Journal of India*.

[27] Devi K., Leondra L., Poovitha R. (2018). A community based study on awareness of organ donation among young adults in rural areas of Puducherry. *International Journal Of Community Medicine And Public Health*.

[28] Srinivasula S., Srilatha A., Doshi D., Reddy B. S., Kulkarni S. (2018). Influence of health education on knowledge, attitude, and practices toward organ donation among dental students. *Journal of Education and Health Promotion*.

[29] Sugumar J., Padhyegurjar M., Padhyegurjar S. (2017). An interventional study on knowledge and attitude regarding organ donation among medical students. *International Journal of Medical Science and Public Health*.

